# Subinhibitory concentrations of resveratrol reduce alpha-hemolysin production in *Staphylococcus aureus* isolates by downregulating *saeRS*

**DOI:** 10.1038/s41426-018-0142-x

**Published:** 2018-07-31

**Authors:** Jingjing Duan, Meilan Li, Zhihao Hao, Xiaofei Shen, Li Liu, Ye Jin, Shanshan Wang, Yinjuan Guo, Lehe Yang, Liangxing Wang, Fangyou Yu

**Affiliations:** 1 Department of Laboratory Medicine, the First Affiliated Hospital of Wenzhou Medical University, Wenzhou, 325000 China; 2 Emergency Intensive Care Unit, Shanghai Pulmonary Hospital, Tongji University School of Medicine, Shanghai, 200082 China; 3 Department of Respiratory Medicine, the First Affiliated Hospital of Wenzhou Medical University, Wenzhou, 325000 China; 4 Department of Laboratory Medicine, Shanghai Pulmonary Hospital, Tongji University School of Medicine, Shanghai, 200082 China; 5 Department of Respiratory Medicine, Affiliated Yueqing Hospital of Wenzhou Medical University, Wenzhou, 325600 China

## Abstract

Resveratrol is a natural phytoalexin. In recent studies, it has been shown to have beneficial effects on cardiovascular disease and cancer and has been deemed to have effective antiviral and immunomodulatory activities. Methicillin-resistant *Staphylococcus aureus* is a multidrug-resistant pathogen associated with skin and soft tissue infections. Alpha-hemolysin is known to play a key role in the symptoms caused by *S. aureus*, and the *saeRS* two-component system has been shown to be a major regulatory system of *S. aureus* virulence. The present study was designed to determine the effect of subinhibitory concentrations of resveratrol on the production of alpha-hemolysin in *S. aureus*. The effect of resveratrol on the transcription of *S. aureus* was studied by transcriptome sequencing. A total of 760 genes with >2-fold changes in expression were selected, including 479 upregulated genes and 281 downregulated genes. On the basis of transcriptome sequencing, the expression of alpha-hemolysin in the *S. aureus* strains of the resveratrol-treated group was downregulated. Our results showed that resveratrol weakly inhibited the growth of *S. aureus* strains, and subinhibitory concentration of resveratrol decreased the expression of *hla* and inhibited the regulation of *saeRS*. Hemolysis testing confirmed that resveratrol had an inhibitory effect on the hemolysis of rabbit erythrocytes infected with *S. aureus* strains in a dose-dependent manner. Resveratrol also decreased the hemolytic capacity by reducing the production of alpha-hemolysin. We found that resveratrol could decrease the expression of *hla* and reduce the secretion of alpha-hemolysin by downregulating *saeRS*. These findings have provided more evidence of the potential of resveratrol as a drug for resisting *S. aureus* infections.

## Introduction

*Staphylococcus aureus* is the main cause of community-acquired bacterial infections and nosocomial infections^1^. A variety of drugs have been used in the treatment of *S. aureus* infection; however, bacterial drug resistance is an increasing problem. In particular, the emergence of methicillin-resistant *S. aureus* strains resistant to most antibiotics is becoming a severe threat to public health, spurring the development of novel antibacterial agents^2^. *S. aureus* can produce a variety of virulence factors, including hemolytic toxins, enterotoxin, coagulase, proteolytic enzymes, and leukotoxin. The virulence of hemolytic toxins, in particular, should not be underestimated. Hemolysin has strong pathogenicity, and its principal types include alpha-hemolysin, beta-hemolysin, gamma-hemolysin, and delta-hemolysin.

Alpha-hemolysin is extremely important and is the most studied pore-forming toxin^3,4^. *S. aureus* alpha-hemolysin (Hla), produced at late logarithmic growth phase, is a 33.2 kDa soluble protein containing 293 amino acid residues and can mediate the death of several different types of cells including erythrocytes, endothelial cells, and an array of immunological cells such as T cells, B cells, and monocytes^5–7^. Hla has a marked hemolytic effect on red blood cells from various mammals, especially rabbit erythrocytes^8^, and plays a significant role in skin and soft tissue infections in animal models of staphylococcal infection. Accordingly, development of drugs targeting hemolysin is a new direction for the treatment of *S. aureus* infection.

Resveratrol (trans-3,4′,5-trihydroxystilbene) is a polyphenolic compound first mentioned in a Japanese article from 1940, where it was isolated from the plant *Veratrum grandiflorum* by root separation^9^. It has subsequently been found in many plants such as mulberry, pomegranate, cranberry, blueberry, and peanut^9,10^. Resveratrol is a natural phytoalexin and has many biochemical activities. Recently, several studies have shown that it not only acts as a plant antitoxin against fungal infections but is also considered a promising multitarget anticancer drug in cancer prevention and treatment^11–13^. Resveratrol is also known to have effective antibacterial activity^14^.

The *saePQRS* system of Staphylococcus aureus controls the expression of major virulence factors and encodes a histidine kinase (SaeS), a response regulator (SaeR), a membrane protein (SaeQ), and a lipoprotein (SaeP)^15^. The *saeRS* system is considered to be a major regulatory system, as the *sae* locus is essential for the transcription of *hla*, *hlb* and *coa*^16^. The *S. aureus* global regulators—*agr, sarA* and *sae*—coordinately control *hla* expression in vitro, and although several distinct regulatory circuits can affect *hla* expression in vitro and in vivo, *sae* appears to play a crucial role^17^. Deletion of *saeRS* resulted in attenuated expression of the genes encoding alpha-hemolysin (*hla*) and the Panton-Valentine leukocidin (*lukSF-PV*) in USA300. Subsequently, the toxin (Hla) was undetectable at any time point after *saeRS* deletion^18^.

In recent years, a new generation of RNA sequencing technology (transcriptome sequencing or RNA-seq) has been widely used in transcriptome studies^19^. RNA-seq has many advantages over microarray analysis. RNA-seq provides excellent genomic coverage and generates over 600 million reads in a single run^20^. Here we applied RNA-seq to investigate the relationship between resveratrol and the metabolism and virulence of *S. aureus* in terms of up- and downregulation of gene expression levels. GO enrichment analysis was used to determine the functional enrichment of differentially expressed genes, and gene metabolic pathways were analyzed using the KEGG system. The analysis of transcriptome sequencing data could provide guidance for further experiments.

In this study, we chose four strains for experimentation. The SA75 strain belongs to ST88, an *S. aureus* strain isolated from an abscess. SA75 has many virulence factors and significant hemolytic activity in phenotype experiments. The USA300 strain belongs to ST8 and has a high prevalence and morbidity rate over a period of time^21^. The MW2 (USA400) epidemic clone has also been the predominant epidemic clone in several Canadian provinces and some parts of the United States^22^. SA759 belongs to ST239, which is a major cause of MRSA infections in Asian hospitals^23^. To prove that resveratrol has universal effects on the hemolytic activity of *S. aureus*, we selected different ST-type *S. aureus* strains for experiments. This study aimed to clarify the influence of resveratrol on the transcriptome of *Staphylococcus aureus* by transcriptome sequencing technology and determine the effect of subinhibitory concentrations of resveratrol on the production of alpha-hemolysin in *S. aureus*. These findings provide more evidence of the potential of resveratrol as a drug for use against *S. aureus* infections.

## Results

### Influence of subinhibitory concentrations of resveratrol on the growth of *S. aureus* strains

The MIC value of resveratrol against *S. aureus* strains was 512 μg/ml. The inhibitory effect of resveratrol on SA75, USA300, MW2, and SA759 was increased with resveratrol drug concentration in a dose-dependent manner. At the subinhibitory concentrations of resveratrol, 1/8 × MIC and 1/16 × MIC, the amount of bacteria at the late logarithmic growth phase was consistent (Fig. 1).

**Fig. 1:** Growth curves of *S.aureus* strains cultured with different concentrations of resveratrol. **a** SA75. **b** USA300. **c**.MW2 **d**.SA759

### Regulation of resveratrol on the main virulence factors of *Staphylococcus aureus*

RNA samples extracted from resveratrol-treated SA75 (SA75 cultured with 1/16 × MIC resveratrol) and untreated SA75 were sequenced on an Illumina HiSeq X platform using a pe150 strategy. The sequencing data were obtained for Res-SA75 (3.3 Gb) and untreated SA75 (3.48 Gb). According to the standard criteria of |log_2_ (fold change)| > 1 and *q* value < 0.005, 760 genes were found to have differential expression (expression difference greater than a 2-fold change), including 479 upregulated genes and 281 downregulated genes (Fig. 2). More importantly, our findings showed that resveratrol can downregulate hemolysin-related genes, including alpha-, gamma- and delta-hemolysin; genes associated with infection such as fibrinogen-binding protein, aggregation factor A, and immunoglobulin-binding protein Sbi; some putative proteins; and genes related to capsular polysaccharide synthesis proteins, such as cap5B, cap8C, cap8F and cap8M (Table 1).

**Fig. 2:** Volcano plot of differences in gene expression between SA75 and Res-SA75. The abscissa refers to the fold-change in the two samples; the ordinate refers to the statistically significant difference in gene expression; red dots indicate a significant difference in upregulated genes and green dots indicate downregulated genes

**Table 1:** This table shows the expression changes of several important genes associated with virulence, capsular polysaccharide synthesis protein, transcription factors, two-component systems, bacterial secretion system, and metabolic function after treatment with resveratrol. The log_2_ (fold-change) indicates the multiples of change of Res_SA75 gene compared to SA75, *p* value is to determine statistically significant indicators, *q* value is the corrected *p* value, and description is based on NCBI annotations for gene description

Gene_id	log_2_ (fold change)	*p* value	*q* value	Description
Virulence				
*MW_RS05590*	−2.572	0.00291	0.00137	fibrinogen-binding protein
*MW_RS04155*	−3.1677	0	0	clumping factor A
*MW_RS01065*	−3.1896	4.36E-16	3.97E-16	hypothetical protein
*MW_RS12680*	−5.0398	9E-130	4.1E-129	immunoglobulin-binding protein sbi
*MW_RS05625*	−2.5486	3.3E-150	1.8E-149	alpha-hemolysin
*MW_RS12700*	−2.1253	2E-09	1.38E-09	gamma-hemolysin component B
*MW_RS11595*	−5.9995	2.3E-243	2.2E-242	toxin
Capsular biosynthesis protein				
*MW_RS00660*	−1.7321	6.17E-05	0.000033	capsular biosynthesis protein
*MW_RS00665*	−1.9846	2.78E-07	1.71E-07	cap5B
* MW_RS00670*	−2.2281	2.42E-08	1.58E-08	cap8C
*MW_RS00685*	−3.5189	2.25E-42	3.83E-42	cap8F
*MW_RS00695*	−3.5263	2.52E-25	3E-25	capsular biosynthesis protein
*MW_RS00720*	−3.1934	1.18E-11	9.06E-12	cap8M
Two-component system				
*MW_RS03395*	1.1992	3.17E-27	3.97E-27	bacitracin ABC transporter permease
*MW_RS03385*	1.0589	1.86E-15	1.66E-15	sensor histidine kinase
*MW_RS13835*	5.4222	1.77E-64	4.2E-64	alkaline phosphatase
*MW_RS06385*	1.1225	3.1E-208	2.3E-207	glutamine synthetase
*MW_RS09935*	1.3879	1.79E-36	2.71E-36	two-component sensor histidine kinase
*MW_RS06850*	7.5208	1.4E-108	5.6E-108	phosphate-binding protein
*MW_RS01260*	−3.7746	2.26E-67	5.47E-67	antiholin-like protein LrgB
*MW_RS03625*	−2.287	1.16E-39	1.85E-39	two-component sensor histidine kinase
*MW_RS05200*	−2.0359	1.66E-07	1.04E-07	cytochrome ubiquinol oxidase subunit I
*MW_RS05355*	−2.0036	1.66E-23	1.86E-23	heme A synthase
*MW_RS01255*	−2.2563	1.51E-05	8.35E-06	murein hydrolase regulator *lrgA*
Transcriptional regulator				
*MW_RS06325*	−2.287	1.16E-39	1.85E-39	*saeS*
*MW_RS03630*	−2.3253	3.32E-24	3.82E-24	*saeR*
*MW_RS00405*	1.1026	7.82E-27	9.66E-27	AraC family transcriptional regulator
*MW_RS03420*	1.4482	6.35E-23	7.02E-23	AraC family transcriptional regulator
*MW_RS12035*	−1.7707	0.010163	0.004536	AraC family transcriptional regulator
*MW_RS13405*	3.5085	6.3E-77	1.71E-76	TetR family transcriptional regulator
*MW_RS13160*	1.0948	2.04E-30	2.74E-30	GntR family transcriptional regulator
*MW_RS05270*	−2.3928	3.3E-07	2.02E-07	Cro/Cl family transcriptional regulator
*MW_RS00880*	−4.002	6.18E-97	2.17E-96	RpiR family transcriptional regulator
*MW_RS01265*	1.3642	1.02E-53	2.08E-53	GntR family transcriptional regulator
*MW_RS01310*	−2.5644	6.91E-17	6.49E-17	LacI family transcriptional regulator
*MW_RS02250*	1.5379	9.93E-10	6.98E-10	LysR family transcriptional regulator
*MW_RS11265*	−1.9478	7.02E-09	4.73E-09	transcriptional regulator
*MW_RS01515*	2.2694	1.09E-66	2.63E-66	transcriptional regulator
*MW_RS03425*	−3.2885	2.6E-70	6.58E-70	transcriptional regulator
*MW_RS13855*	−4.0504	2.6E-36	3.89E-36	transcriptional regulator

### Effect of a subinhibitory concentration of resveratrol on *hla* expression

To verify the relative expression levels of *hla* (the gene encoding alpha-hemolysin) and *saeRS* (the locus regulating *hla*) of *S. aureus* strains after incubation with resveratrol, real-time RT-PCR was performed. We found that increasing concentrations of resveratrol significantly reduced transcription of *hla* and *saeRS* in these strains. According to the results of transcriptome sequencing, the expression of *saeR* was downregulated after adding resveratrol, which was consistent with the RT-PCR results. After culturing strains with resveratrol (1/8 × MIC) for 16 h, *hla* expression was decreased by 11.9-fold (*P* < 0.01) to 1.73-fold (*P* < 0.01) compared with that of the untreated group; *saeR* was decreased by 17.4-fold (*P* < 0.01) to 2.02-fold (*P* < 0.01), and the transcription of *saeS* was consistent with that of *saeR*. These results inferred that resveratrol can reduce the hemolytic capacity of *S. aureus* strains by inhibiting expression of *hla*, especially in SA759 (Fig. 3).

**Fig. 3:** Relative expression of *hla* and *saeR/S* in *S.aureus* strains after cultured with various concentrations of resveratrol. Values are means + SDs (based on three repeated assays). There were significant differences with the control group (grown without resveratrol) for each strain (*P* < 0.05)

### Effect of resveratrol on the hemolytic activity of *S. aureus* strains

The effect of resveratrol on alpha-hemolysin in *S. aureus* culture supernatants was assessed using hemolysin assays with the percentage of hemolysis obtained by comparison with the untreated group. Resveratrol treatment depressed the activity of alpha-hemolysin in culture supernatants. The hemolysis activity of the experimental group without drug treatment was significantly higher than that of groups treated with different concentrations of resveratrol (from 1/16 × MIC to 1/4 × MIC). When cultured with 1/16 × MIC resveratrol, 4.63–34.16% of the rabbit erythrocytes were lysed by alpha-hemolysin. When cultured in 1/8 × MIC resveratrol, hemolysis percentages decreased to 1.9–8.15%. The results showed that hemolytic activity decreased with increasing drug concentration in a concentration-dependent manner (Fig. 4).

**Fig. 4:** Effect of resveratrol on the hemolytic activity of *S.aureus* strains. There were significant differences with the control group (grown without resveratrol) for each strain (*P* < 0.05). Each test was performed independently in triplicate

### Influence of resveratrol on alpha-hemolysin in *S. aureus* culture supernatants

According to *hla* gene expression analysis and hemolysin assays, we needed to verify the effect of resveratrol on alpha-hemolysin expression at the protein level. The results of many experiments showed that there was no significant difference between the untreated group and the 1/16 × MIC group for the concentration of alpha-hemolysin determined by ELISA (P > 0.05), so we chose 1/8 × MIC to conduct the following experiment. At the 1/8 × MIC concentration of resveratrol, the concentrations of alpha-hemolysin in the four strains were 10.28 pg/ml (SA75), 7.46 pg/ml (USA 300), 9.66 pg/ml (MW2), and 10.92 pg/ml (SA759), while those in untreated groups were 19.25 pg/ml, 11.11 pg/ml, 16.77 pg/ml and 22.19 pg/ml, respectively. These results showed that the production of alpha-hemolysin was markedly reduced by resveratrol treatment at 1/8 × MIC (Fig. 5), which was consistent with the findings of the previous hemolysis phenotype assays.

**Fig. 5:** Effects of a sub-inhibitory concentration of resveratrol on alpha-hemolysin (Hla) release was quantified by ELISA in *S.aureus* strains grown with or without resveratrol. The test was performed independently in triplicate

### Influence of subinhibitory concentrations of resveratrol in a skin infection model

To determine the influence of resveratrol on the virulence of *S. aureus*, 4- to 6-week-old BALB/C-nu mice were subcutaneously injected with 1.0 × 10^7^ CFU/100 µl SA75. The mice were divided into the wild-type group administered SA75 not exposed to resveratrol and the SA75-treated group, which was treated with SA75 cultured with 1/8 MIC Res. The resulting abscess sizes in mice inoculated in the treated group were smaller than the lesion sizes in animals infected in the wild-type group. The lesions remained until the end point of the experiment. As shown in Fig. 6, animals challenged with 1.0 × 10^7^ CFU/100 μl SA75 had significantly larger (*P* < 0.05) skin lesions than animals challenged with an equivalent amount of SA75 in the treated group. These data demonstrated that resveratrol could indeed weaken the virulence of *S. aureus*.

**Fig. 6:** Results of mouse skin infection model experiments. **a** Comparison of abscess size (area) of SA75 wild-type group and SA75-treated-group (cultured with 1/8 MIC Res). **b** Skin lesions resulting from S. aureus infection (picture taken at day 2 of infection)

## Discussion

*Staphylococcus aureus* is becoming one of the most important human pathogens due to its strong resistance to drugs and the prevalence of multidrug-resistant strains in hospitals. The continuing emergence of multidrug-resistant strains of *S. aureus* from nosocomial and community sources is becoming a public health problem. On the basis of transcriptome sequencing results, we concluded that resveratrol can impact the expression of multiple *Staphylococcus aureus* genes, and the subinhibitory concentration of resveratrol could attenuate the virulence of *Staphylococcus aureus* by affecting the expression of virulence factors. In our experiments, we found that resveratrol could reduce alpha-hemolysin secreted by *Staphylococcus aureus* by downregulating *saeRS*.

Bacterial drug resistance arises through a variety of mechanisms, from alterations in the protein targets of antimicrobial agents to changes in metabolic pathways to the production of antibiotic-inactivating enzymes^24,25^. Various antimicrobial agents are being developed considering the corresponding bacterial resistance mechanisms. Vancomycin and linezolid are common drugs currently used against MRSA infections, and they are also the last significant line of defense against MRSA. As *Staphylococcus aureus* resistance gradually increases, however, the effectiveness of these drugs continuously decreases^26^. In addition to drug resistance, virulence factors produced by MRSA are also important in infectious diseases. Such virulence factors include leukotoxin, protease, capsular polysaccharide, and hemolysin and are directly or indirectly involved in infections caused by *S. aureus*. Consequently, development of agents targeting *S. aureus* virulence factors is a promising approach for the treatment of *S. aureus*-induced infections. In this study, the experimental results showed that subinhibitory concentrations of resveratrol reduced the hemolytic capacity of *S. aureus*.

Resveratrol has a variety of biological activities including anticancer activity, immune regulation, prevention of cardiovascular disease, antioxidation and antiviral effects. The mechanism of its antibacterial effect, however, is not clear. Paulo *et al*. found that resveratrol has antibacterial activity against a variety of bacteria; the antibacterial activity of resveratrol is greater against gram-positive bacteria than against gram-negative bacteria^14^. In this experiment, we selected four strains of different ST-type *S. aureus* strains and found that high concentrations of resveratrol had inhibitory effects on bacterial growth, and the MIC value of resveratrol against these *S. aureus* strains was 512 μg/ml. We further explored the effect of resveratrol on *S. aureus* virulence factors and found that it could inhibit the expression of *hla*. Alpha-hemolysin is a well-characterized and prominent virulence factors in severe infections caused by *S. aureus*, especially those involving methicillin-resistant strains. Alpha-hemolysin is the first bacterial exotoxin to be identified as a pore former, and it plays a significant role in the skin and soft tissue infections models caused by *S. aureus*. Many studies have shown that some chemical inhibitors and drugs can significantly inhibit the virulence of *S. aureus* by inhibiting the transcription or function of *hla*^8^. In our study, resveratrol was shown to reduce the hemolytic capacity of *S. aureus* by inhibiting the expression of transcriptional regulatory genes such as *saeR, saeS* and *hla*. It has been found that alpha-hemolysin production can be controlled at either the transcriptional (by *saeRS*, and, to a lesser extent, by *agr*) or the translational (by *agr*) level by these global regulators^27^. The roles of *saeP* and *saeQ* are less well defined; they likely act to modulate *saeRS* expression, but *saeP* may also have an independent regulatory function^28^. In our experiment, comparing transcriptome data from the untreated group with that of the resveratrol-treated group indicated that expression of the transcription factor *saeRS* was downregulated with increased concentrations of resveratrol. RT-PCR results verified that the expression of *saeRS* did indeed decrease. However, the expression of *saePQ* did not show concentration-dependent results. We thus deduced that the effect of resveratrol on alpha-hemolysin depends on *saeRS* as an independent regulation system that regulates alpha-hemolysin by downregulating *saeRS*. Our results indicated that resveratrol may potentially act on *S. aureus* virulence factors.

In this study, to investigate the effects of subinhibitory concentrations of resveratrol on *S. aureus*, we studied the growth of *S. aureus* strains, performed transcriptome analysis of its metabolic pathways, analyzed differential expression of genes following treatment with resveratrol, and studied the regulation of alpha-hemolysin and its mechanism of action. Our aim was to understand the molecular mechanism of pathogenicity, virulence and metabolism of *S. aureus* strains under the action of resveratrol, a Chinese herbal medicinal compound. According to the transcriptome sequencing results, the important virulence factor, alpha-hemolysin, was downregulated, and the regulation of *saeRS* was also downregulated. Real-time qPCR showed that *saeR/S* gene expression decreased with increasing concentrations of resveratrol. It was speculated that the regulation of resveratrol on alpha-hemolysin depended on *saeRS*, and *saeRS* regulated the expression of *hla*. According to hemolysis testing, we found that hemolytic activity of *S. aureus* decreased with increasing drug concentration. ELISA was used to detect the expression of alpha-hemolysin at the protein level, and the results were consistent with the phenotypic results, which showed that resveratrol could downregulate the expression of alpha-hemolysin and inhibit hemolytic activity. The experiment using a mouse abscess model also confirmed that resveratrol could indeed weaken the virulence of *Staphylococcus aureus*. The data reported here also provide a basis for exploring potential drug targets and developing new drugs to treat *Staphylococcus aureus* infections.

## Materials and methods

### Bacterial strains and reagents

The strains used in the experiments were SA75, USA300, MW2, and SA759. Resveratrol (3,4′,5-trihydroxistilbene) was purchased from Sigma-Aldrich (St. Louis, MO, USA). The resveratrol solution used in the experiments was dissolved in dimethyl sulfoxide (DMSO, BOYUN, SH, China). All reagents used were of analytical grade.

### Determination of the MIC of resveratrol

Different concentrations of resveratrol were prepared in DMSO. The broth microdilution method based on CLSI guidelines was used to determine the minimal inhibitory concentration (MIC)^29^. The MIC was defined as the lowest concentration at which no visible growth was observed. *S. aureus* ATCC 29213 was used as the control strain in accordance with CLSI breakpoints.

### Growth assay

The *S. aureus* strains were grown in TSB (BD, NJ, USA) to an optical density (OD) value of 0.3 at 600 nm, and the cultures were aliquoted into five flasks. Varying doses of resveratrol was added to three of the cultures to obtain final concentrations of 1/16, 1/8 and 1/4 × MIC (32, 64 and 128 µg/ml, respectively). One of the cultures received 1% DMSO only to verify whether DMSO affects bacterial growth. The 5th flask was a control culture that contained TSB only. All cultures were incubated at 37 °C with shaking at 220 rpm, and the OD600 value was measured every hour for 24 h and used to draw growth curves.

### RNA-seq and identification of differentially expressed genes

Strains were cultured in TSB with added resveratrol at 37 °C. After 16 h, the bacteria were collected for the extraction of total RNA by centrifugation at 4 °C for 2 min at 12,000 rpm. Total RNA was extracted using QIAGEN RNeasy Maxi columns according to the manufacturer’s instructions (QIAGEN, Berlin, Germany). Qualitative RNA samples were analyzed by RNA-seq (transcriptome sequencing) using an Illumina HiSeq X platform and the pe150 (150 bp double-stranded assay) strategy. Sequencing data from the SA75 and RES-SA75 (SA75 cultured with 1/16 × MIC of resveratrol) samples were analyzed using DEGseq software to determine the effect of resveratrol on gene expression. The screening of differential genes mainly included the multiple and significant level of gene expression. It was generally considered that |log_2_ (Fold Change)| > 1 and *P* < 0.005 indicated differences in gene expression between samples.

### Real-time RT-PCR

Strains were cultured in TSB to which different concentrations of resveratrol were added at 37 °C. RNA was extracted according to the method described earlier. The primer pairs used in real-time RT-PCR are listed in Table 2. The cDNA was synthesized from total RNA using a Takara RNA PCR kit (Takara, Tokyo, Japan) according to the manufacturer’s instructions. PCRs were performed in 20 µl reaction mixtures using Luna Universal qPCR Master Mix (NEB, MA, USA). Each test was performed independently in triplicate.

**Table 2:** Primers used for real-time RT-PCR

Primer name	Sequence (5′ → 3′)
*gyrb*-RT-F	ACATTACAGCAGCGTATTAG
*gyrb*-RT-R	CTCATAGTGATAGGAGTCTTCT
*hla*-RT-F	TGGTAATCATCACGAACTC
*hla*-RT-R	GCAGCAGATAACTTCCTT
*saeR*-RT-F	GTCGTAACCATTAACTTCTG
*saeR*-RT-R	ATCGTGGATGATGAACAA
*saeS*-RT-F	TGTATTTAAAGTGATAATATGAGTC
*saeS*-RT-R	CTTAGCCCATGATTTAAAAACACC

### Hemolysis assay

Hemolysis assays were used to determine the inhibitory effect of resveratrol on the release of alpha-hemolysin. Strains were cultured in TSB at 37 °C with shaking at 220 r.p.m., and different concentrations of resveratrol were added to the culture medium. After 16 h, bacteria were collected from cultures and adjusted to the same OD (OD600 nm = 2.5). Bacterial samples (1 ml) were centrifuged (5500 × *g*, 4 °C, 1 min), the resulting supernatants were filtered with a 0.22-µm filter, and 0.1 ml of supernatant was brought up to 975 µl with PBS. After incubation with 25 µl defibrinated rabbit blood for 1 h at 37 °C, the samples were centrifuged (5500 ×*g*, room temperature, 1 min) and the OD of the supernatants was measured at 600 nm. Triton X-100 was used as a positive control, and 0.01 M PBS was used as a negative control. Each test was performed independently in triplicate.

### Enzyme-Linked Immunosorbent Assay (ELISA) for Alpha-Hemolysin

*S. aureus* strains were cultured in 1/8 × MIC resveratrol-treated TSB, 1/16 × MIC resveratrol-treated TSB and untreated TSB, respectively. Bacterial supernatants were extracted as described previously. Purified staphylococcal alpha-hemolysin antibody (Sigma-Aldrich, St. Louis, MO, USA) was used to coat microtiter plate wells, and different supernatants were then added to the wells. When the staphylococcal alpha-hemolysin antibody was combined with the HRP label, these mixtures became an antibody-antigen-enzyme labeled antibody complex. After washing completely, TMB (3,3′,5,5′-tetramethylbenzidine) substrate solution was added, the reaction was terminated by the addition of a sulfuric acid solution, and the color change was measured spectrophotometrically at a wavelength of 450 nm. The concentration of alpha-hemolysin in the samples was then determined by comparing the OD of the samples to the standard curve. We considered the standard density to be the horizontal axis, and the OD value was the vertical axis. The standard curve was drawn, and a straight line regression equation for the standard curve with the standard density was calculated. According to the equation, we calculated the sample density, multiplied by the dilution factor, and determined the actual concentration of alpha-hemolysin. Each test was performed independently in triplicate.

### Mouse model of skin abscess infection

Animal studies were approved by the Institutional Animal Care and Use Committee. We confirmed that all animal care and methods were performed in accordance with the guidelines and regulations approved by the Administration of Affairs Concerning Experimental Animals in China. The skin abscess model was performed as described^30^. Male 4- to 6-week-old BALB/C-nu mice were used in the study. The mice were housed for 7 days with food and water before inoculation. SA75 was cultured in 1/8 × MIC resveratrol-treated TSB and untreated TSB, respectively. *S. aureus* cultures were grown to the postexponential phase, washed with sterile phosphate-buffered saline (PBS), and then suspended in PBS to achieve a concentration of 1.0 × 10^7^ CFU/100 µl. The bacterial numbers were confirmed by plate counts. After the mice were anesthetized with diethyl ether, each mouse was injected subcutaneously with 100 µl of either *S. aureus* suspension or PBS. Skin lesions were observed daily, and the abscesses were measured. The abscess area was calculated using the formula *A* *=* *π* (*L* *×* *W*) / 2, where *L* is the length and *W* is the width. The values of *L* and *W* for each infected mouse were determined by caliper. Abscesses were observed and recorded for 7 days, after which all animals were killed.

### Statistical analysis

Experimental data were analyzed using GraphPad Prism 6 software (version 6.00, La Jolla, CA, United States). A *p* value less than 0.05 was considered to be statistically significant.
